This article has been retracted.

# Inhibitory Effect of Ursolic Acid on Proliferation and Migration of Renal Carcinoma Cells and Its Mechanism

**DOI:** 10.1155/2022/1529132

**Published:** 2022-05-04

**Authors:** Xiao Lyu, Xuhui Zhang, Libin Sun, Jingqi Wang, Dongwen Wang

**Affiliations:** ^1^Department of Urology, First Hospital of Shanxi Medical University, Taiyuan 030001, Shanxi, China; ^2^First College of Clinical Medicine, Shanxi Medical University, Taiyuan 030001, Shanxi, China; ^3^National Cancer Center/National Clinical Research Center for Cancer/Cancer Hospital and Shenzhen Hospital, Chinese Academy of Medical Sciences and Peking Union Medical College, Shenzhen 518100, Guangdong, China

## Abstract

**Background:**

Renal carcinoma is one of the most common malignant tumors in the urinary system. Autophagy can be both activated and inhibited in renal carcinoma, and it plays a double-edged role in the development of renal carcinoma. In the early stage of cancer, autophagy can suppress tumors. In the late stage, autophagy contributes to the survival of tumor cells in an unfavorable environment, and some autophagy-related proteins P62, LC3B, and beclin-1 have become indicators of the prognosis of patients with renal carcinoma.

**Aim:**

To demonstrate that ursolic acid activates autophagy in renal carcinoma 786-O cells by inhibiting the hedgehog signaling pathway.

**Methods:**

The effect of ursolic acid on the viability of 786-O cells was determined by the MTT method; the effect of ursolic acid on the proliferation and migration of 786-O cells was examined by crystalline violet staining and scratch assay, respectively. For the study of autophagy, we firstly screened the time points. Western blot assay was used to detect the expression level of autophagic protein P62 at different time points of ursolic acid on 786-O. Then, the Cell ^MeterTM^ Autophagy Assay Kit was used to detect the effect of different doses of ursolic acid on the autophagic fluorescence intensity of 786-O cells; the Western blot method was used to detect the effect of different doses of ursolic acid on the expression levels of LC3II and P62 proteins in 786-O cells. Further, AdPlus-mCherry-GFP-LC3B adenovirus transfection was used to detect the effect of ursolic acid on the autophagic flow of 786-O cells; ursolic acid was combined with the autophagy inhibitor chloroquine (CQ) to detect the expression level of autophagy protein LC3II by Western blot. In terms of mechanism, the effect of ursolic acid on hedgehog signaling pathway-related proteins in 786-O cells was detected by Western blot.

**Results:**

Ursolic acid inhibited the activity, proliferation, and migration of 786-O cells, enhanced the fluorescence intensity of autophagosomes in 786-O cells, increased the expression level of autophagy marker protein LC3II, and inhibited the expression level of P62 in a time and dose-dependent manner; ursolic acid activated the autophagic flow in 786-O cells, which showed that ursolic acid caused the accumulation of autophagic fluorescent spots and enhanced the fluorescence intensity of autophagosomes. Ursolic acid activated the autophagic flow in 786-O cells, as evidenced by the accumulation of autophagic fluorescent spots and enhanced fluorescence intensity of autophagosomes, and the combined use of the autophagy inhibitor CQ increased the expression level of LC3II compared to ursolic acid alone; ursolic acid decreased the expression levels of PTCH1, GLI1, SMO, SHH, and c-Myc and increased the expression level of Sufu in the hedgehog signaling pathway.

**Conclusion:**

Ursolic acid activates autophagy in renal carcinoma 786-O cells, probably by inhibiting hedgehog signaling pathway activity.

## 1. Introduction

Renal carcinoma is one of the most common cancers is one of the most common malignant tumors in the urinary system [1]. By 2030, the number of new cases is expected to exceed 2.2 million and the number of deaths will exceed 1.1 million [2]. Hedgehog signaling pathway plays an important role in the growth and differentiation of human tissues and is critical for the body to maintain homeostasis in a physiological state [3]. Activation of the hedgehog signaling pathway involves multiple molecular components [4]. When the Hh ligand binds to PTCH1, a typical receptor for SMO inhibition, it leads to SMO aggregation and phosphorylation, which induces the segregation of downstream GLI1 proteins from Sufu and then into the nucleus to induce transcription of a range of oncogenes [5]. Most studies have shown that aberrant activation of the hedgehog signaling pathway is associated with the development, progression, and recurrence of renal carcinoma [6]. Autophagy is a highly evolutionarily conserved process that occurs when cellular contents, including damaged proteins, organelles, etc., are transferred to lysosomes and digested and degraded by enzymes for recycling [7]. When cells are exposed to unfavorable environments, such as nutrient deficiency, the mammalian target of rapamycin (mTOR) will be inhibited, followed by activation of the ULK complex (FIP200, Atg13, ULK) and then the downstream PI3KIII complex (hvps34, beclin-1, p150, UVRAG) to induce autophagy. Atg12-Atg5 and Atg7-Atg3, two interconnected systems, play an important role in the extension of autophagic membranes to form autophagosomes and their fusion with lysosomes to form autophagic lysosomes to disassemble their contents. Recent studies have shown that autophagy is closely associated with aberrant activation of the hedgehog signaling pathway. In this study, we investigated whether ursolic acid could regulate the proliferation, migration, and autophagy of renal carcinoma 786-O cells. For the study of autophagy, we firstly screened the time points. Western blot assay was used to detect the expression level of autophagic protein P62 at different time points of ursolic acid on 786-O. Then, the Cell ^MeterTM^ Autophagy Assay Kit was used to detect the effect of different doses of ursolic acid on the autophagic fluorescence intensity of 786-O cells; the Western blot method was used to detect the effect of different doses of ursolic acid on the expression levels of LC3II and P62 proteins in 786-O cells. Also, we further explored whether its mechanism was related to its inhibition of hedgehog signaling pathway activity to provide an experimental basis for the search for new anti-renal carcinoma active ingredients from traditional Chinese medicine.

## 2. Materials and Methods

### 2.1. Materials

Renal carcinoma cell line 786-O was purchased from the Shanghai Cell Bank, Chinese Academy of Sciences. The sources of reagent instruments used in this study are as follows: Ursolic acid (Chengdu Manstead Biotechnology Co., Ltd., Lot No. MUST-17070501); GANT61 (Sigma-Aldrich, Lot No. 21798); MyCoy5A medium (Beijing Wokawei Biotechnology Co., Ltd., Lot No. AF29530969); Fetal bovine serum (Beijing Sai Aomei Cell Technology Co. 20180524); RIPA lysate (Hubei Dr.D. Biological Co., Ltd., Lot No. 15E28C05); Protease inhibitor (Lot No. P1010-1), AdPlusmCherry-GFP-LC3B adenovirus (Lot No. C3012), 4% paraformaldehyde (Lot No. 1808573), crystalline violet (Lot No. C0121) (Shanghai Ltd.); GLI1 (Beijing Biosun Biotechnology Co., Ltd., Lot No. A103296468); SHH (Lot No. 20697-1-AP), Sufu (Lot No. 26759-2-AP) (Wuhan Sanying Biotechnology Co., Ltd.); PTCH1 (Immunoway Inc., Lot No. YT3598); c Myc (Chengdu Zhengneng Biotechnology Co., Ltd., Lot No. 20190313); SMO (Hangzhou Hua'an Biotechnology Co., Ltd., Lot No. HN0716); GAPDH primary antibody (Lot No. A00131), HRP-labeled sheep anti-rabbit IgG secondary antibody (Lot No. YR202912) (Hangzhou Unitech Biotechnology Co., Ltd.); P62 (Lot No. 39749), LC3 (lot 12741) (CST, USA); Cell MeterTM Autophagy Assay Kit (AAT, USA, lot 23000);CO2 incubator (Thermo, USA, model Forma3111); Ultra-clean bench (Suzhou Antai Air Technology Co., Ltd, model SW-CJ-2FD); Confocal microscope (Leica GmbH, Germany, model SP8SR); Bio-Rad gel imaging system (Burroughs Corporation, USA, model 721BR11389).

### 2.2. Methodology

#### 2.2.1. Effect of Ursolic Acid on the Viability of 786-O Cells Measured by MTT Method

786-O cells in the logarithmic growth phase were inoculated in 6-well plates at 5 000 cells per well, and the cell-free wells were set as zeroing wells. After about 8 h, the original medium was discarded and a series of drug-containing medium containing different concentrations of ursolic acid (90, 60, 45, 30, 15, and 7.5 ^*μ*mol−L−1^) was added. After 24 h of incubation, 10 *μ*L of MTT working solution was added to each well and incubated at 37°C with 5% _CO2_ for 4 h. The liquid in the wells was discarded and DMSO (150 *μ*L/well) was added. After incubation, the absorbance (A) at 570 nm was measured by ELISA, and the cell survival rate and _IC50_ were calculated. Cell survival rate = (*A*_administered wells_ − *A*_zeroed wells_)/(*A*_normal wells_ − A _zeroed wells_) × 100%.

#### 2.2.2. Effect of Ursolic Acid on the Proliferation of 786-O as Detected by Crystalline Violet Staining

786-O cells in good growth condition were digested and inoculated with 1 000 cells per well in 6-well plates, and the culture was continued for 7 d. The medium was changed every 2 d. The medium was discarded, and a medium containing different doses of ursolic acid (20, 10, 5 *μ*mol-L-1) and GANT61 (20 *μ*mol-L-1) was added. The medium was discarded, and a medium containing different doses of ursolic acid (20, 10, 5 ^*μ*mol−L−1^) and GANT61 (20 ^*μ*mol−L−1^) were added. After 72 h of action, the original medium was discarded, 4% paraformaldehyde was fixed for 15 min, and the crystalline violet staining solution was added for 10 min and then washed three times with PBS to observe the effect of drugs on the proliferation of 786-O cells.

#### 2.2.3. Scratch Test for the Effect of Ursolic Acid on the Migration of 786-O

After trypsin digestion, 786-O cells were collected and inoculated in 24-well plates (1 × ^105^ cells/well), and when the monolayer of cells spread across the bottom of the plate, a cross was crossed with a 10-*μ*L gun, washed with PBS, and drug-containing medium containing different doses of ursolic acid (20, 10, 5 ^*μ*mol−L−1^) and GANT61 (20 ^*μ*mol−L−1^) was added immediately. Then, photographs were taken under an inverted microscope at 0, 12, and 24 h. The healing area was measured by ImageJ, and the percentage of wound healing was calculated.

#### 2.2.4. Selection of Autophagy Time Points

1. Cell ^MeterTM^ Autophagy Assay Kit was used to detect the number of autophagosomes at different time points. 786-O cells at logarithmic growth stage were inoculated in 96-well plates (5 000 cells/well) at 5 time points (0, 4, 8, 12, and 24 h). After about 8 h, the old medium was discarded and 200 *μ*L of ursolic acid at a concentration of 20 ^*μ*mol−L−1^ was added at different time points, and then the old medium was discarded. The autophagy fluorescence intensity was observed by inverted fluorescence microscopy.
2. Western blot method is to detect the expression level of autophagy protein P62 at different time points. 786-O cells were inoculated in 6-well plates at 6×10^5^ cells/well, and after cell apposition, 2 mL of ursolic acid at a concentration of 20 *μ*mol-L-1 was administered at 4, 8, 12, and 24 h, respectively. Cells were collected, total cell protein was lysed, and protein concentration was determined by the BCA method. The protein concentration was determined by the BCA method. A certain amount of loading buffer was added according sample volume, denatured at high temperature and then electrophoresed, blocked by 5% BSA for 90 min, and the primary antibody was washed three times for 5 min each time in TBST.

#### 2.2.5. Cell ^MeterTM^ Autophagy Assay Kit Detects the Effect of Different Doses of Ursolic Acid on the Autophagosome of 786-O Cells

786-O cell suspensions in logarithmic growth phase were collected and inoculated in 30 mm confocal dishes at ^1×104^ cells/well. After about 8 h, the old medium was discarded, 1 mL of medium was given to the blank group, and ursolic acid (20, 10, 5 ^*μ*mol−L−1^) and GANT61 (20 ^*μ*mol−L−1^) were given to each group with corresponding doses of drug-containing medium, and the old medium was discarded after 24 h. Each well was washed once with 500 *μ*L of PBS, and 100 *μ*L of LCell ^MeterTM Autophagy Assay Kit^ was added. Then, the cell was incubated for 30 min at 37 °C and observed with a Leica confocal microscope. Fluorescence images were taken with a 630x oil microscope, and the fluorescence intensity of each image was analyzed using ImageJ software.

#### 2.2.6. Effect of Ursolic Acid on Autophagic Flow in 786-O Cells

1. AdPlus-mCherry-GFP-LC3B adenovirus transfection assay to detect the effect of ursolic acid on autophagic flow in 786-O cells. 30 mm laser copolymer dishes were submerged in filtered 100 ^*μ*g-mL−1^ poly-D-lysine (PLL) solution for 5 min and then placed in an ultra-clean table with open air blowing and UV sterilization. 786-O cells in logarithmic growth phase were inoculated with ^2×104^ cells per well in 30 mm laser copolymer dishes. The cells were incubated in a _CO2_ incubator (5% _CO2_, 37°C), and adenovirus transfection was performed when the fusion level of the cells was 50% under the microscope in the laser confocal dish. The cells in each dish were infected with mCherry-GFP-LC3B adenovirus solution (MOI = 40) for 24 h. The adenovirus solution was discarded, and the cells were continued to be cultured for 24 h. The successful transfection was observed under an inverted fluorescence microscope. After the adenovirus solution was discarded, the normal group was given 1 mL (0.1% DMSO) of complete medium, and ursolic acid (20, 10, 5 *μ*mol−L_−1_) was given 1 mL of drug-containing medium in each group.
2. Combination of ursolic acid and the autophagy inhibitor chloroquine (CQ) to detect the expression level of the autophagy protein LC3II by Western blot.

786-O cells were inoculated in ^6×105^ cells/well in 6-well plates, and after the cells were fused to about 40%, ursolic acid high-dose group (20 ^*μ*mol−L−1^), GANT61 group (20 ^*μ*mol−L−1^), ursolic acid high-dose (20 ^*μ*mol−L−1^) + CQ (25 ^*μ*mol−L−1^) group, GANT61 (20 ^*μ*mol−L−1^) + CQ (^25 *μ*mol−L−1^) group, and blank control group were set up. ^1^) +CQ (25 ^*μ*mol−L−1^) group, CQ group (25 ^*μ*mol−L−1^), and blank control group. The drug-containing medium was washed once with PBS, and the wells were incubated with the corresponding drug-containing medium for 24 h. Western blot was then performed as described above, and the protein bands were analyzed by Image Lab after completion.

#### 2.2.7. Western Blot Assay to Detect the Effect of Ursolic Acid on the Expression Levels of Hedgehog Signaling Pathway and Autophagy Proteins in 786-O Cells

786-O cells were inoculated at ^6×105^ cells/well in a 6-well plate, and the cells were fused to about 40% and given medium containing ursolic acid (20, 10, 5 ^*μ*mol−L−1^) and GANT61 (20 ^*μ*mol−L−1^) at different concentrations, respectively. The protein bands were analyzed by Image Lab.

### 2.3. Statistical Analysis

The data were analyzed by SPSS 19.0 statistical software, and the experimental data were expressed as mean ± standard deviation ( $\bar{x}\pm s$). *t*-Test was used for comparison between two groups, and one-way ANOVA was used for comparison between multiple groups. <0.05 indicates that the difference is statistically significant.

## 3. Results

### 3.1. Inhibition of 786-O Activity by Ursolic Acid In Vitro

Compared with the solvent control, different doses of ursolic acid (90, 60, 45, 30, and 15 ^*μ*mol−L−1^) significantly inhibited 786-O cell activity (*p* < 0.01), and the inhibitory effect increased with higher doses of ursolic acid (Table 1).

### 3.2. Ursolic Acid Inhibits the Proliferation of 786-O Cells

The high dose of ursolic acid (20 *μ*mol/L) and the GANT61 (20 *μ*mol/L) group almost completely inhibited the clonal growth of 786-O cells, followed by the medium dose of ursolic acid (10 *μ*mol/L) and to a lesser extent the low dose (5 *μ*mol/L) group (Figure 1).

C, solvent control group; P, GANT61 20 ^*μ*mol−L−1^ group; L, ursolic acid 5 ^*μ*mol−L−1^ group; M, ursolic acid 10 ^*μ*mol−L−1^ group; H, ursolic acid 20 ^*μ*mol−L−1^ group (notations are similar for Figures 2–5).

### 3.3. Ursolic Acid Inhibits Migration of 786-O Cells

Compared with the solvent control group, the GANT61 group and ursolic acid high (20 *μ*mol/L) and medium (10 *μ*mol/L) dose groups could inhibit the migration of 786-O cells at 12 and 24 h (*p* < 0.01 or *p* < 0.05); compared with 12 h, the GANT61 (20 *μ*mol/L) group and ursolic acid at different doses (20, 10, 5) could inhibit the migration of 786-O cells at 24 h (*p* < 0.01). The inhibition of migration of 786-O cells was more obvious in the GANT61 (20 *μ*mol-L-1) and ursolic acid groups (20, 10, 5 ^*μ*mol−L−1^) at 24 h. The difference was statistically significant (*p* < 0.01) (Figure 2).

### 3.4. Autophagy Induction by Ursolic Acid in 786-O Cells

Compared with the solvent control group, the ursolic acid high-dose group was able to inhibit the expression of the autophagy-related protein P62 at the time point of 24 h (Figure 6) (*p* < 0.05) (Figure 3). Therefore, the autophagy time point was set at 24 h for the subsequent experiments.

### 3.5. Enhanced Autophagosome Fluorescence of 786-O Cells by Ursolic Acid

Compared with the solvent control group, the GANT61 (20 *μ*mol/L) group and ursolic acid high (20 *μ*mol/L) and medium (10 *μ*mol/L) dose groups enhanced the fluorescence intensity of autophagosomes in 786-O cells (*p* < 0.01 or *P* < 0.05), and unlike the solvent control group, which showed diffuse and weak fluorescence, the above groups could be seen as aggregates with enhanced fluorescence. The fluorescence of autophagosomes was enhanced in the above groups, suggesting that autophagy was activated (Figure 3).

### 3.6. Activation of 786-O Cellular Autophagic Flow by Ursolic Acid

Compared with the solvent control group, yellow fluorescent spots were clustered in the GANT61 (20 *μ*mol/L) group and ursolic acid high (20 *μ*mol/L), medium (10 *μ*mol/L), and low (5 *μ*mol/L) dose groups, and red fluorescent spots increased with increasing ursolic acid dose, suggesting that autophagic processes were not blocked and autophagic flow was activated; the autophagy late inhibitor CQ inhibited the degradation of LC3II (*p* < 0.05), and the expression level of LC3II was elevated in the ursolic acid high dose (20 *μ*mol/L) and GANT61 (20 *μ*mol/L) groups (*p* < 0.05); after CQ was combined with ursolic acid and GANT61, the expression of LC3II was increased compared with that before the combination (*p* < 0.05), indicating that ursolic acid and GANT61 activated autophagosome formation rather than inhibiting autophagosome degradation (Figure 4).

### 3.7. Ursolic Acid Inhibited Hedgehog Signaling Pathway Activity to Activate Autophagy Compared with the Solvent Control Group

Medium (10 *μ*mol/L) and low (5 *μ*mol/L) dose groups significantly inhibited the expression of the pathway protein PTCH1 (*P* < 0.01 or *P* < 0.05); the GANT61 (20 *μ*mol/L) group and the ursolic acid high (20 *μ*mol/L) and medium (10 *μ*mol/L) dose groups increased the expression of LC3II, a marker protein of autophag (*P* < 0.01 or *P* < 0.05), while the expression level of P62 was significantly decreased (*P* < 0.01) (Figure 6).

## 4. Discussion

Renal carcinoma is one of the most common malignant tumors in the urinary system. Recent studies have shown that autophagy is closely associated with aberrant activation of the hedgehog signaling pathway. Autophagy can be both activated and inhibited in renal carcinoma, and it plays a double-edged role in the development of renal carcinoma [8, 9]; in the early stage of cancer, autophagy can suppress tumors, while in the late stage, autophagy contributes to the survival of tumor cells in an unfavorable environment, and some autophagy-related proteins P62, LC3B, and beclin-1 have become indicators of the prognosis of patients with renal carcinoma [10, 11]. Autophagy is a dynamically changing process [12, 13], and this experiment was conducted to map the autophagy time point, and the results showed that the activation of autophagy was more obvious when ursolic acid acted on 786-O cells at 24 h. Therefore, the time point of the subsequent experiment was set to 24 h. It was found that ursolic acid could increase the expression level of LC3II protein in 786-O cells, which is considered as autophagy. However, the reason for this may be the increased autophagosome production and also the blocked degradation phase of autophagosomes, so the degradation phase was inhibited using the autophagic tool drug CQ in combination to observe whether the expression level of LC3II was changed [14]. AdPlus-mCherry-GFP-LC3B adenovirus was also used to transfect cells, based on the principle that in the case of non-autophagy, mCherry-GFP-LC3B is present in the cytoplasm as diffuse yellow fluorescence under fluorescence microscopy, In the case of autophagy, mCherry-GFP-LC3B aggregated on the autophagosome membrane under fluorescence microscope, presenting as yellow spots; When the autophagosome and lysosome fuse, they appear as red spots due to partial quenching of GFP fluorescence. The above experimental results suggest that ursolic acid and GANT61 activate the autophagosome formation phase, but do not inhibit the lysosome fusion degradation phase [15, 16]. Currently, hedgehog pathway inhibitors have been widely used as a treatment for various types of cancers caused by pathway overactivation.

## 5. Conclusion

The present experimental study showed that ursolic acid, a novel inhibitor of hedgehog signaling pathway, could induce autophagy in renal carcinoma cells 786-O (Figure 7), but since the role of autophagy in renal carcinoma remains controversial, whether it will promote or prevent renal carcinoma progression remains to be further investigated. Our future research direction is to analyze the effect of autophagy cells on carcinoma.

## Figures and Tables

**Figure 1:** Effect of ursolic acid on the proliferation of 786-O cells.

**Figure 2:** Effect of ursolic acid on the migration of 786-O cells. *p* < 0.05 compared with solvent control; ^*∗*^*p* < 0;01; ^*∗∗*^*p* < 0.01; ^##^*p* < 0.01 compared with 12 h.

**Figure 3:** Effect of ursolic acid on autophagy in 786-O cells.

**Figure 4:** Effect of ursolic acid on autophagic flow in786-O cells. Notes: CQ, chloroquine 25 *μ*mol·L^−1^ group; P+CQ. GANT61 20 *μ*mol·L^−1^ + chloroquine 25 *μ*mol·L^−1^ group; H+CQ. ursolic acid 20 *μ*mol·L^−1^ + chloroquine 25 *μ*mol·L^−1^ group; 2 groups compared, ^#^*P* < 0.05.

**Figure 5:** Effect of ursolic acid on the expression of hedgehog signaling pathway proteins and autophagy-related proteins.

**Figure 6:** Effect of ursolic acid on autophagy of 786-O cells at different time points. ^*∗*^*p*  < 0.05 compared with 0 h.

**Figure 7:** Ursolic acid activates 786-O cell autophagy by inhibiting the hedgehog signaling pathway.

**Table 1:** Effect of ursolic acid on the activity of 786-O cells ($\bar{x}\pm s$, *n* = 6).

Ursolic acid (*μ*mol/L)	A570 nm
0	0.82 ± 0.12
90	0.13 ± 0.02^1)^
60	0.16 ± 0.03^1)^
45	0.20 ± 0.05^1)^
30	0.31 ± 0.10^1)^
15	0.48 ± 0.08^1)^
7.5	0.68 ± 0.13

Note: ^1)^refers to compared to solvent control, *P* < 0.01.

## Data Availability

The datasets used and/or analyzed during the current study are available from the corresponding author on reasonable request.

## References

[1] Park B. J., Seaman S. C., Noeller J. L. (2021). Metastatic Renal Cell Carcinoma to the Spine: Outcomes and Morbidity: Single-Center Experience. *World Neurosurgery*.

[2] Khene Z. E., Mathieu R., Peyronnet B. (2021). Radiomics can predict tumour response in patients treated with Nivolumab for a metastatic renal cell carcinoma: an artificial intelligence concept. *World Journal of Urology*.

[3] Rosiello G., Palumbo C., Knipper S. (2021). Comparison of survival outcomes in patients with metastatic papillary vs. clear-cell renal cell carcinoma: a propensity-score analysis. *World Journal of Urology*.

[4] Li Q., Li N., Luo Y. (2020). Role of intraoperative ultrasound in robotic-assisted radical nephrectomy with inferior vena cava thrombectomy in renal cell carcinoma. *World Journal of Urology*.

[5] Tsuruoka C., Kaminishi M., Shinagawa M. (2021). High relative biological effectiveness of 2 MeV fast neutrons for induction of medulloblastoma in Ptch1+/- mice with radiation-specific deletion on chromosome 13. *Radiation Research*.

[6] Bai J.-Y., Jin B., Ma J.-B. (2021). HOTAIR and androgen receptor synergistically increase GLI2 transcription to promote tumor angiogenesis and cancer stemness in renal cell carcinoma. *Cancer Letters*.

[7] Mandhair H. K., Arambasic M., Novak U., Radpour R. (2020). Molecular modulation of autophagy: new venture to target resistant cancer stem cells. *World Journal of Stem Cells*.

[8] Chhabra R., Nanjundan M. (2020). Lysophosphatidic acid reverses Temsirolimus-induced changes in lipid droplets and mitochondrial networks in renal cancer cells. *PLoS One*.

[9] Wang S., Jia M., Su M. (2020). Ufmylation is activated in renal cancer and is not associated with von Hippel-lindau mutation. *DNA and Cell Biology*.

[10] Wang X., Jiang Y., Zhu L. (2020). Autophagy protects PC12 cells against deoxynivalenol toxicity via the Class III PI3K/beclin 1/Bcl‐2 pathway. *Journal of Cellular Physiology*.

[11] Pavlinov I., Salkovski M., Aldrich L. N. (2020). Beclin 1-atg14l protein-protein interaction inhibitor selectively inhibits autophagy through disruption of VPS34 complex I. *Journal of the American Chemical Society*.

[12] Sun X., Wang Z., Shao C. (2021). Analysis of chicken macrophage functions and gene expressions following infectious bronchitis virus M41 infection. *Veterinary Research*.

[13] Deng M., Zhang G., Cai Y. (2020). DNA methylation dynamics during zygotic genome activation in goat. *Theriogenology*.

[14] Vega-Rubín-de-Celis S., Kinch L., Peña-Llopis S. (2020). Regulation of beclin 1-mediated autophagy by oncogenic tyrosine kinases. *International Journal of Molecular Sciences*.

[15] Borah A., Pillai S. C., Rochani A. K. (2020). GANT61 and curcumin-loaded PLGA nanoparticles for GLI1 and PI3K/Akt-mediated inhibition in breast adenocarcinoma. *Nanotechnology*.

[16] Zhang Z., Zhang R., Hao C., Pei X., Li J., Wang L. (2020). GANT61 and valproic acid synergistically inhibited multiple myeloma cell proliferation via hedgehog signaling pathway. *Medical Science Monitor : International Medical Journal of Experimental and Clinical Research*.

